This article has been retracted.

# MicroRNA‐92a promotes tumor growth and suppresses immune function through activation of MAPK/ERK signaling pathway by inhibiting PTEN in mice bearing U14 cervical cancer

**DOI:** 10.1002/cam4.1329

**Published:** 2018-05-11

**Authors:** Zeng‐Hui Li, Lei Li, Lin‐Ping Kang, Yan Wang

**Affiliations:** ^1^ Department of Obstetrics and Gynecology The Affiliated Yantai Yuhuangding Hospital of Qingdao University Yantai 264000 China; ^2^ Department of Obstetrics and Gynecology Qingdao Municipal Hospital Qingdao 266071 China; ^3^ Department of Obstetrics The Affiliated Yantai Yuhuangding Hospital of Qingdao University Yantai 264000 P.R. China

**Keywords:** Immune function, MAPK/ERK signaling pathway, MicroRNA‐92a, PTEN, U14 cervical cancer

## Abstract

Cervical cancer is known as the possible outcome of genital infection, while the molecular mechanisms of initiation, development, and metastasis of cervical cancer have not yet been fully elucidated. Our study aims to investigate the effects of microRNA‐92a (miR‐92a) on tumor growth and immune function by targeting PTEN *via* the MAPK/ERK signaling pathway in tumor‐bearing mice. C57BL/6 female mice were used for tumor‐bearing mouse models and their tumor and adjacent normal tissues were collected, and normal cervical tissues were obtained from normal mice. Serum levels of tumor necrosis factor‐*α* (TNF‐*α*) and soluble interleukin‐2 receptor (sIL‐2R) were detected by ELISA. The cells were divided into the normal, blank, negative control (NC), miR‐92a mimic, miR‐92a inhibitor, siRNA‐PTEN, and miR‐92a inhibitor + siRNA‐PTEN groups. Dual‐luciferase reporter assay was adopted to determine the relationship between PTEN and miR‐92a. Expressions of miR‐92a, PTEN, TNF‐*α*, sIL‐2R, ERK1, and ERK2 were tested by RT‐qPCR and Western blotting. Cell proliferation was detected by cell count kit‐8 **(** CCK‐8); cell cycle and apoptosis were detected by flow cytometry. Compared with the normal cervical tissues and adjacent normal tissues, the cervical cancer tissues exhibited increased expressions of miR‐92a, p‐ERK1/2, and serum levels of TNF‐*α* and sIL‐2R while decreased PTEN expression. PTEN was confirmed to be the target gene of miR‐92a. As compared with the blank and NC groups, expressions of miR‐92a, ERK1 and ERK2 increased, and expressions of PTEN decreased in the miR‐92a mimic group. The miR‐92a mimic group exhibited increased expression levels of TNF‐*α* and sIL‐2R, cell proliferation, and cell number in S phase but decreased cell apoptosis, and cell number in G0/G1 phase, while the miR‐92a inhibitor group followed opposite trends. miR‐92a promotes tumor growth and suppresses immune function by inhibiting PTEN *via* activation of the MAPK/ERK signaling pathway in mice bearing U14 cervical cancer.

## Introduction

Cervical cancer is considered to be the second most prevalent malignant tumor that greatly threatens women's health, predominantly arising from the infection of the high‐risk subtypes of human papilloma virus (HPV) 1, 2. It was estimated that approximately 500,000 new cases and more than 250,000 deaths are caused by cervical cancer across the world, and in China, the number of incident case was predicated to reach 93,000 in 2030, and the mortality rate was especially high in rural China 3. Cervical cancer screening and various treatment programs are well applied in therapies, but they have not reached optimum implementation in developing countries 4. Granted that cervical cancer at early stages can be treated by conventional therapies, later period cervical cancer is untreatable with low survival 5. Fortunately, microRNAs (miRNAs) have been identified to play an important role in cancer pathogenesis by regulating molecular aberration or gene expression, which suggested the possible use of it as an anticancer therapy 6.

MiRNAs, a subset of short noncoding RNAs (17–22 nucleotides), could post‐transcriptionally regulate the expression of relevant genes and thus participate in the development of cervical cancer 7. Approximately, 70 miRNAs have been discovered to be involved in cervical cancer thus far and the list is ever growing 8. MicroRNA‐92a (miR‐92a), which belongs to the family of miR‐17‐92, has been evidenced to be responsible for the onset and progression of various common human cancers, including pancreatic cancer 9. PTEN is a tumor‐suppressed gene, and the inability of PTEN may be essential in the pathogenesis of various human malignancies, including cervical cancer 10. It has been indicated that the MAPK signaling pathway may be responsible for the inhibition of expression and functioning of PTEN 11. Repression of MAPK signaling pathway has similar effects on the maintenance of PTEN, which revealed that the MAPK signaling pathway leads to the restoration of advanced breast cancers harboring PTEN loss 12. Mitogenic‐activated protein kinase (MAPK)/extracellular signal‐regulated kinase (ERK) signaling pathway has been found to play a role in some cancer therapies, as ERK1/2, one of MAPK/ERK kinases, was highly expressed in cervical cancer tissues 13, which also regulates many biological factors that affect types of miRNAs and their relevant machinery 14. It has been indicated that some miRNAs, like miR‐22, might have potential effects on cell biology via the regulation of PTEN expression 15. Tumor necrosis factor‐alpha (TNF‐*α*) is involved in the restoration of immune homeostasis, as proinflammatory cytokine 16. However, the targeting mechanism of miR‐92a on PTEN affecting cervical cancer via the MAPK/ERK signaling pathway remains to be elucidated. In our study, we aim to explore the ability of miR‐92a to regulate the progression of U14 cervical cancer cell by targeting PTEN *via* the MAPK/ERK signaling pathway, in order to provide a novel therapeutic target for cervical cancer.

## Materials and Methods

### Tumor‐bearing mouse model establishment

C57BL/6 clean‐grade female mice (18–22 g) in closed group were provided by the Animal Laboratory, Nanjing General Hospital of Chinese PLA Nanjing Military Region. All mice were housed in plastic boxes with regular cleaning under controlled conditions of temperature (20 ± 2°C), relative humidity illumination (8–10 h), and free access to feed (man‐made) and water. U14 cervical cancer cell line of mice was purchased from the Shanghai Institute of Material Medical (Shanghai, China). U14 was seeded in the C57BL/6 mice, and the ascites was preserved followed by passaging. Mice bearing U14 cervical cancer that were passaged for 10 days were treated with injections of ascites. After the abdomen skin was disinfected, the milk‐white ascites was extracted *via* a sterile injector, and the tumor cell density was adjusted to 1 × 10^7^ cells/mL using normal saline. Right subaxillary skin was disinfected and then inoculated with 0.2 mL of U14 cervical cancer cell suspension for the establishment of tumor‐bearing mouse models. After 15 days of feeding, cancer tissues (*n *= 40) and adjacent tissues (*n *= 20) were extracted. At the same period, normal cervical tissues (*n *= 15) of normal mouse were collected under sterile conditions after execution. A portion of these extracted tissues were placed in liquid nitrogen for the extraction of RNA and proteins, and the rest were preserved in paraformaldehyde for the preparation of paraffin sections. All experiment processes for mice were in accordance with the ethical standard for animal treatment, and all efforts were made to minimize the number of animals used and their suffering.

### Immunocytochemistry

Streptavidin–peroxidase (SP) method was used for immunohistochemical staining, of which immunohistochemical kit and Diaminobenzidine (DAB) chromogenic agent were both purchased from Beijing Zhongshan Biotechnology Company (Beijing, China). The samples were embedded in paraffin conventionally and sliced into 4 *μ*m thick serial sections. After routine dewaxing and gradient hydration, endogenous peroxidase was blocked by 3% hydrogen peroxide and antigen, and was repaired by microwave. Following the addition of primary mouse anti‐human PTEN monoclonal antibody, the samples were stored at 4°C in a refrigerator overnight. Polymerase adjuvant was added to the samples for incubation at room temperature for 20 min, and horseradish peroxidase (HRP)‐labeled secondary goat anti‐mouse immunoglobulin G‐fluorescein isothiocyanate (IgG‐FITC) (Bioss Antibodies Co., Ltd., Beijing, China) was also added to the samples for incubation at room temperature for 30 min. And then, SP compound was added to the samples for incubation for 20–30 min. The samples were stained with DAB, restained with hematoxylin and mounted. Phosphate buffer saline (PBS) was used as the negative control (NC), with the known U14 cervical cancer samples as the positive control. The PTEN‐positive expression was presented in the cytoplasm with dark brown staining. If bulky colored particles were observed, the position was verified as strong positive (+++), brown and thin colored particles as medium‐strong positive (++), light yellow and no obvious colored particles as positive (+), and no colored particles as negative (−) 17. The positive rate was calculated and recorded.

### Enzyme‐linked immunosorbent assay (ELISA)

ELISA was adopted in order to determine the contents of tumor necrosis factor‐*α* (TNF‐*α*) and soluble interleukin‐2 receptor (sIL‐2R) in mouse serum and transfected cells. Blood (1 mL) was extracted from the eyeball, rested on ice for 30 min, centrifuged for 10 min at 1134 g, and the serum obtained in the supernatant was used for detection of expressions of TNF‐*α* and sIL‐2R. The antigen was dissolved by 50 nmol/L carbonates‐coated buffer solutions (pH 9.6) (concentration of antigen of 10–20 *μ*g/mL) and then added to the 96‐well ELISA plates with 100 *μ*L in each well, which was incubated at 4°C overnight. The next day, the coating liquid was removed prior to phosphate buffer saline tween (PBST) rinsing (three times), and 150 *μ*L of 1% bovine serum albumin (BSA) was added to the wells for 1 h sealing at 37°C. Following PBST rinsing (three times), 100 *μ*L of serum of distinct dilution and sample controls were added to each well for incubation at 37°C for 2 h. And then, 100 *μ*L diluted HRP‐labeled goat anti‐mouse second antibody was added to incubate for 1 h at 37°C. After further PBST rinsing (five times), chromogenic agent was applied for 20‐min coloration. Optical density (OD) value at A450 was obtained in a microplate reader (TECAN‐F50; TECAN, Maennedorf, Switzerland).

### Cell transfection and grouping

Cells were extracted from tissues of cervical cancer model mice and normal control mice, respectively. Cells were assigned into the normal group (epithelial cells in mouse uterus of normal controls), the blank group (no transfection for tumor cells in mouse models), the negative control group (NC group, tumor cells of mouse model transfected with miR‐92a NC sequence), the miR‐92a mimic group (tumor cells of mouse models transfected with miR‐92a mimic sequence), the miR‐92a inhibitor group (tumor cells of mouse models transfected with miR‐92a inhibitor sequence), the siRNA‐PTEN group (tumor cells of mouse models transfected with siRNA‐PTEN sequence), and the miR‐92a inhibitor + siRNA‐PTEN group (tumor cells of mouse models cotransfected with miR‐92a inhibitor sequence and siRNA‐PTEN sequence). All mentioned sequences were synthetized by the Shanghai Sangon Biological Engineering Technology & Services Co., Ltd. (Shanghai, China). The day prior to transfection, the cells were processed for passage and inoculated in a six‐well plates (2 × 10^6^ cells per well). On the day of transfection, the cells reached a confluency of 70–80%. According to the instruments of LiPofectamine^®^ 2000 kit (11668019; Invitrogen Inc., Carlsbad, CA), 250 *μ*L of serum‐free culture medium Opti‐MEM (Gibco Co., Grand Island, NY) was used to dilute 100 pmol miR‐92a inhibitor, miR‐92a mimic, miR‐92a inhibitor + siRNA‐PTEN, siRNA‐PTEN, normal control, blank control and NC (the final concentration was 50 nmol/L), and then the above was mixed and incubated at room temperature for 5 min, respectively. Next, 250 *μ*L of serum‐free culture medium Opti‐MEM was used to dilute 5 *μ*L lipofectamine 2000, and the above was mixed and incubated at room temperature for 5 min. The above two mixtures were mixed, incubated for 20 min at room temperature, and added to the culture wells. After 6 h of transfection, the complete medium was replaced, and the cells were cultured at 37°C in a humidified incubator containing 5% CO_2_ with air for 24–48 h for further experiments.

### Reverse transcription quantitative polymerase chain reaction (RT‐qPCR)

Total RNA of cervical cancer cells and tumors was extracted based on the Trizol method (Invitrogen Inc.) in order to determine the concentration and purity of RNA. The OD260/OD280 values of samples were detected by the ultraviolet spectrophotometer (Shanghai Modern Science Instrument Co., Ltd., Shanghai, China), and RNA concentration was also calculated. The extracted RNA was preserved at −80°C for further use. According to the instructions of the reverse transcription cDNA Kit TaqMan MicroRNA Assays Reverse Transcription Primer (4366596; Thermo scientific, Waltham, MA), the obtained reverse transcription products were diluted by sterile water (diluted at a ratio of 1: 5), followed by preservation at −20°C for further use. The miR‐92a and PTEN primers were synthetized by the Shanghai Biowing Applied Biotechnology Co., Ltd. (Shanghai, China) (Table 1). A total of 20 *μ*L of PCR reaction system were designed as follows: 10 *μ*L of 2 × A11‐in‐One Q‐PCR Mix, 2 *μ*L of All‐in‐One miRNA Q‐PCR Primer (2 *μ*mol/L), 2 *μ*L of Universal Adaptor PCR Primer (2 *μ*mol/L), 2 *μ*L of Cdna (diluted 1:5), 0.4 *μ*L of 50× Rox Reference Dye and 20 *μ*L of DNase/RNase‐free H_2_O. The amplification conditions involved predenaturation at 95°C for 10 min, 40 cycles of denaturation at 95°C for 10 s, annealing at 60°C for 20 s, and elongation at 72°C for 34 s. ABI7500 quantitative PCR (ABI Company, Oyster Bay, NY) was used for RT‐qPCR. U6 was regarded as the internal reference for miR‐92a and *β*‐actin for PTEN. The 2^−ΔΔCt^ method was applied to calculate the relative expressions of target genes.

**Table 1:** Primer sequences for RT‐qPCR

Genes	Primer sequences
miR‐92a	F: 5′‐CACCTATATTGCACTTGTCC‐3′
	R: 5′‐TGCGTGTCGTGGAGTC‐3′
U6	F: 5′‐ACCCTGAGAAATACCCTCACAT‐3′
	R: 5′‐GACGACTGAGCCCCTGATG‐3′
PTEN	F: 5′‐TGGATTCGACTTAGACTTGACCT‐3′
	R: 5′‐GCGGTGTCATAATGTCTCTCAG‐3′
*β*‐actin	F: 5′‐GTGACGTTGACATCCGTAAAGA‐3′
	R: 5′‐GCCGGACTCATCGTACTCC‐3′
ERK1	F: 5′‐TCCGCCATGAGAATGTTATAGGC‐3′
	R: 5′‐GGTGGTGTTGATAAGCAGATTGG‐3′
ERK2	F: 5′‐GGTTGTTCCCAAATGCTGACT‐3′
	R: 5′‐CAACTTCAATCCTCTTGTGAGGG‐3′
TNF‐*α*
	F: 5′‐ATGAGCACTGAAAGCATGATCCGG‐3′
R: 5′‐GCAATGATCCCAAAGTAGACCTGCCC‐3′
sIL‐2R
	F: 5′‐GAATTTATCATTTCGTGGTGGTCTCCG‐3′
R: 5′‐TCTTCTACTCTTCCTCTGTCTCCG‐3′

RT‐qPCR, reverse transcription quantitative polymerase chain reaction; F, forward; R, reverse; miR‐92a, microRNA‐92a; PTEN, phosphatase and tensin homolog deleted on chromosome ten; ERK1, extracellular regulated protein kinases 1; ERK2, extracellular regulated protein kinases 2.

### Western blotting

Proteins were extracted from cells and tumor tissues and used in order to determine the protein concentration according to the instructions of the Bicinchoninic Acid (BCA) Kit (No: P23227; Pierce Chemical, Rockford, IL), and protein concentration was adjusted for all proteins. The extracted protein was quantified, and subsequently, 5× sulfate‐polyacrylamide gel electrophoresis (SDS‐PAGE) loading buffers were added, and protein denaturation was performed at 95°C for 5 min and then SDS‐PAGE was conducted. The samples were electrophoresed using a SDS‐PAGE, transferred to a membrane and blocked using 5% skim milk at 4°C freezer overnight. The membrane was rinsed with tris‐buffered saline tween (TBST), and primary mouse‐antibodies, namely PTEN antibody (CST, Danvers, MA), ERK1 antibody (CST), ERK2 antibody (CST), and p‐ERK antibody (ab214362; Abcam, Cambridge, UK), were added for incubation overnight. Subsequently, the samples were rinsed in TBST supplemented with a horseradish peroxidase (HRP)‐conjugated secondary antibody and cultured for 1 h at 37°C. After rinsing the membrane in TBST, enhanced chemiluminescence (ECL) was employed in order to develop HRP. After developing, the film was extracted, washed by pure water, dried, and recorded. *β*‐actin was used as the internal control; the ratio of gray value between target protein bands and internal control bands was regarded as the relative expression levels.

### Dual‐luciferase reporter assay

The target gene of miR‐92a was predicted with the assistance of biological prediction website TargetScan. The dual‐luciferase reporter gene assay demonstrated that PTEN was the direct target of miR‐92a. Dual‐luciferase reporter assay was used for further identification. The full‐length 3’ untranslated region (UTR) of PTEN was cloned and amplified. The PCR products were subcloned and inserted into the pMirGlo Dual‐Luciferase vector (Promega Corporation, Madison, WI) downstream of the luciferase gene, named as PTEN‐wide type (PTEN‐wt). Next, site‐directed mutagenesis was conducted for the binding site of miR‐92a and its target gene predicted by bioinformatics in order to construct a PTEN‐mutant (PTEN‐mut) carrier. The pRL‐TK carrier expressing renilla luciferase (Takara Holdings Inc., Kyoto, Japan) was adopted as internal control to adjust the distinction of cell quantity and transfection efficiency. The miR‐92a mimic and NC were respectively cotransfected with luciferase reporter carrier into U14 cervical cancer cells, and dual‐luciferase activity was detected by Promega‐provided methods.

### Flow cytometry

Cells were collected 48 h after transfection and digested using a 0.25% trypsin solution, rinsed thrice with cold PBS, and centrifuged with the supernatant eliminated. The collected cells were resuspended with addition of PBS (2 mL for 1 mL cells), and cell concentration was adjusted to 1 × 10^5^ cells/mL. The cells were fixed with 1 mL precooled ethanol solution (−20°C) with a volume fraction of 75% at 4°C for 1 h. The cells were centrifuged again in order to remove the alcohol and then rinsed with PBS twice and the supernatant was discarded. After that, the cells were added with 100 *μ*L of RNase in dark conditions, water‐bathed for 30 min at 37°C, and added with 400 *μ*L of propidium iodide (PI, Sigma‐Aldrich Chemical Company, St Louis, MO) for reaction for 30 min at 4°C. Flow cytometry (EPICS XL, Becton, Dickinson and Company, NJ, US) excited at 488 nm was adopted to record the cell cycle for red fluorescence. Three samples were provided for each group, and each experiment was carried out three times.

After 48 h of transfection, the cells were digested using ethylene diamine tetraacetic acid (EDTA)‐free trypsin, collected in a flow tube, and centrifuged with the supernatant removed. After precooled PBS rinsing three times, the cells were centrifuged with the supernatant discarded again. According to the instructions of Annexin‐V‐FITC cell apoptosis kit (C1065; Beyotime Biotechnology Co., Shanghai, China), Annexin‐V‐FITC, PI, and hydroxyethylpiperazine ethane sulfonic acid (HEPES) buffer solution were used to prepare the Annexin‐V‐FITC/PI staining solution at the ratio of 1: 2: 50. And, 1 × 10^6^ cells were resuspended within every 100 *μ*L of staining solution. After the solution was mixed, the cells were incubated for 15 min at room temperature and mixed again following the addition of 1 mL of HEPES. A 488 nm wavelength was used for the excitation of 525 and 620 nm bands pass filter in order to detect the cell apoptosis by measurement of FITC and PI fluorescence. Three samples were provided for each group, and every experiment was repeated three times.

### Cell countkit‐8 (CCK‐8) assay

The cells were seeded in a 96‐well plates after 48 h of transfection. Six duplicated wells were set for each group, and the total volume of each well was 100 *μ*L (1 × 10^5^cells in each well). The plate was then placed in humidified incubator at 37°C with 5% CO_2_. The OD value was recorded after 0 h, 24 h, 36 h, 48 h, 60 h, and 72 h of culture. The cell activity graph was drawn with the x‐axis referring to time and the y‐axis representing OD value.

### Transplanted tumor

After mice bearing U14 cervical cancer for 27 days, the diameter of a majority of transplanted tumors reached 7–10 mm, and 30 C57BL/6 nude mice were assigned to six groups with five mice in each group as follows: the blank group (no transfection), the NC group (transfected with miR‐92a NC sequence), the miR‐92a mimic group (transfected with miR‐92a mimic sequence), the miR‐92a inhibitor group (transfected with miR‐92a inhibitor sequence), the siRNA‐PTEN group (transfected with siRNA‐PTEN sequence), and the miR‐92a inhibitor + siRNA‐PTEN group (transfected both with miR‐92a inhibitor sequence and siRNA‐PTEN sequence). It should be noticed that the needle was inserted into the tumor from appendant skin and ran under the skin for a while before the needle was inserted into tumor. The drug was injected into several locations in the same tumor with a small amount being injected each time. After that, the injection was repeated once every 3 days with a total of six times. The tumor growth and size were observed at the 0th day, 3rd day, 6th day, 9th day, 12th day, and 15th day, respectively.

### Statistical analysis

Statistical analyses were performed using the SPSS 18.0 (SPSS Inc., Chicago, IL). Counting data among groups were compared using the chi‐squared test, and measurement data were presented as mean ± standard deviation (SD). If the recorded data were normally distributed and had homogeneous variance, *t*‐tests were used for comparisons between two groups and one‐way analysis of variance (ANOVA) was used for comparisons among multiple groups. Spearman's rank correlated method was adopted for correlation analysis. *P *<* *0.05 was considered to be statistically significant.

## Results

### Positive expression rate of PTEN protein is lowest in cervical cancer tissues

According to immunohistochemistry results, PTEN was predominantly found in the cytoplasm presented as dark brown grain coloration. The positive expression rate of PTEN was 37.5% in cervical cancer tissues and 70.0% in adjacent normal tissues. However, the positive expression rate of PTEN reached 100% in normal cervical tissues, suggesting that the expression rate decreased with increasing malignant degree of cancer (*P *<* *0.05) (Fig. 1, Table 2). In conclusion, highest levels of positive expression rate of PTEN were observed in the normal cervical tissues while lowest in cervical cancer tissues.

**Figure 1:** Positive expression rate of PTEN in normal cervical tissues, adjacent normal tissues, and cervical cancer tissues (SP, 200×). PTEN, phosphatase and tensin homolog deleted on chromosome ten; SP, streptavidin–peroxidase.

**Table 2:** Positive expression rate of PTEN protein the cervical cancer tissues, adjacent normal tissues, and normal cervical tissues

Groups	Numbers	Expressive intensity of PTEN				Ratio of positive expression (%)
		**−**	+	++	+++	
Normal cervical tissues	15	0	8	4	3	100
Adjacent normal tissues	20	6	5	6	3	70*
Cervical cancer tissues	40	25	10	4	1	37.5*#

*P <* *0.05 compared with the normal cervical tissues. #*P *<* *0.05 compared with the adjacent normal tissues; PTEN, phosphatase and tensin homolog deleted on chromosome ten.

### TNF‐*α* and sIL‐2R are expressed at highest levels in mouse serum of cervical cancer tissues

According to ELISA results, higher levels of TNF‐*α* and sIL‐2R were found in mouse serum in the cervical cancer and adjacent normal tissues compared to the normal cervical tissues. Cervical cancer tissues also exhibited higher levels of TNF‐*α* and sIL‐2R compared to the adjacent normal tissues (all *P *<* *0.05) (Table 3). In summary, TNF‐*α* and sIL‐2R are highly expressed in mouse serum of cervical cancer tissues.

**Table 3:** Serum levels of sIL‐2R and TNF‐*α* in three groups

Groups	Numbers	Cell factors	
		sIL‐2R (U/mL)	TNF‐*α* (pg/mL)
Normal cervical tissues	15	155.3 ± 50.25	186.6 ± 76.13
Adjacent normal tissues	20	239.32 ± 83.08*	256.49 ± 93.37*
Cervical cancer tissues	40	356.02 ± 143.18*, #	391.64 ± 161.0*, #

*P <* *0.05, compared with the normal cervical tissues; ^#^ *P *<* *0.05, compared with the adjacent normal tissues; TNF‐*α*, tumor necrosis factor‐*α*; sIL‐2R, soluble interleukin‐2 receptor.

### MiR‐92a, TNF‐*α*, sIL‐2R, ERK1, and ERK2 are overexpressed and PTEN is underexpressed in cervical cancer tissues

According to the RT‐qPCR and Western blotting results (Fig. 2), the expression of miR‐92a, mRNA and protein expressions of ERK1, ERK2, TNF‐*α*, and sIL‐2R were found to be increased in the cervical cancer tissues compared to the adjacent normal tissues and normal cervical tissues, while mRNA and protein expression of PTEN were comparatively diminished (all *P *<* *0.05). In cervical cancer tissues, the protein expression of PTEN presented a lower level in comparison with the adjacent normal and normal cervical tissues, whereas ERK1, ERK2, p‐ERK1, and p‐ERK2 proteins were highly expressed, as opposed to the adjacent normal and normal cervical tissues. Besides, the ratio of p‐ERK1/ERK1 and p‐ERK2/ERK2 was significantly higher than the adjacent normal and normal cervical tissues (all *P *<* *0.05). Taken together, expressions of miR‐92a, ERK1, ERK2, TNF‐*α*, and sIL‐2R showed a higher level while expression of PTEN presented a lower level in cervical cancer tissues.

**Figure 2:** MiR‐92a expression, mRNA and protein expressions of PTEN, TNF‐*α* and sIL‐2R expressions, and ERK1/2 in normal cervical tissues, adjacent normal tissues and cervical cancer tissues. (A) miR‐92a expression, mRNA expressions of PTEN and ERK1/2; (B) Western blotting map; (C) protein gray value of PTEN and ERK1/2; miR‐92a, microRNA‐92a; PTEN, phosphatase and tensin homolog deleted on chromosome ten; ERK1/2, extracellular regulated protein kinases 1/2; *, *P *<* *0.05 compared with the normal cervical tissues and adjacent normal tissues

### PTEN is verified as the target gene of miR‐92a

The miRNA online software TargetScan predicted the presence of binding sites between PTEN and miR‐92a (Fig. 3A). To verify PTEN as one of the direct target genes of miR‐92a, the wild (PTEN‐wt) and mutant (PTEN‐mut) sequences lacking miR‐92a combination sites in PTEN 3'UTR area were inserted into the reporter plasmid. The miR‐92a mimic and PTEN‐wt or PTEN‐mut recombined plasmid were cotransfected into the U14 cervical cancer cells using luciferase activity assay, and the results showed that miR‐92a mimic had no significant effects on the luciferase activity of PTEN‐mut, while that of the PTEN‐wt group decreased by 43% (*P *<* *0.05) (Fig. 3B). These findings indicate that miR‐92a may suppress luciferase activity of PTEN‐wt plasmid. In addition, PTEN is the potential target gene of miR‐92a.

**Figure 3:** PTEN is determined as a target gene of miR‐92a. (A) predicted binding sites of miR‐92a at PTEN 3′UTR; (B) detection of luciferase activity; miR‐92a, microRNA‐92a; PTEN, phosphatase and tensin homolog deleted on chromosome ten; *, *P *<* *0.05, compared with the NC group.

### Overexpressed miR‐92a decreases PTEN expression, and increases TNF‐*α*, sIL‐2R, ERK1, and ERK2 expressions

RT‐qPCR and Western blotting were adopted in order to assess miR‐92a expression and mRNA and protein expressions of PTEN, TNF‐*α*, sIL‐2R, and related genes in the MAPK/ERK after cell transfection in seven groups. There were no significant differences in terms of miR‐92a expression, mRNA, and protein expressions of PTEN, ERK1, ERK2, p‐ERK1, p‐ERK2, TNF‐*α*, and sIL‐2R between the blank and NC groups (*P *>* *0.05). Compared with the normal group, miR‐92a expressed higher in the rest groups. In contrast to the blank and NC groups, the expression of miR‐92a and expressions of ERK1, ERK2, TNF‐*α*, sIL‐2R, p‐ERK1, and p‐ERK2 were increased, with the activation of MAPK/ERK signaling pathway, and the mRNA, and protein expressions of PTEN decreased in the miR‐92a mimic group, while the miR‐92a inhibitor showed opposite trends (all *P *<* *0.05). In comparison with the blank and NC groups, mRNA and protein expressions of PTEN decreased, and mRNA and protein expressions of TNF‐*α*, sIL‐2R, p‐ERK1, p‐ERK2, ERK1, and ERK2 increased in the siRNA‐PTEN group. No significant differences were found in miR‐92a expression and mRNA and protein expressions of PTEN, ERK1, ERK2, TNF‐*α*, sIL‐2R, p‐ERK1 and p‐ERK2 between the blank and NC groups and the miR‐92a inhibitor + siRNA‐PTEN group (all *P *>* *0.05) (Fig. 4 and Table A1). These findings provide evidence that overexpression of miR‐92a increased mRNA and protein expressions of ERK1, ERK2, TNF‐*α*, sIL‐2R, p‐ERK1 and p‐ERK2 and decreased mRNA and protein expressions of PTEN.

**Figure 4:** MiR‐92a expression and mRNA and protein expression of PTEN, TNF‐*α*, sIL‐2R and ERK1/2 in seven groups after transfection. A, miR‐92a expression, mRNA expression of PTEN, TNF‐*α*, sIL‐2R and ERK1/2; B, Western blotting map; C, protein gray value of PTEN and ERK1/2; miR‐92a, microRNA‐92a; PTEN, phosphatase and tensin homolog deleted on chromosome ten; ERK1/2, extracellular regulated protein kinases 1/2; *, *P *<* *0.05 compared with the normal group; ^#^, *P *<* *0.05 compared with the blank and negative control groups.

### MiR‐92a promotes cell proliferation in vitro

The results of CCK‐8 assay showed that the OD value at every time point was of no significance between the miR‐92a mimic group and the siRNA‐PTEN group (*P *>* *0.05), and both of the two groups marked higher OD values at 72 h and 96 h compared to the blank and NC groups, suggesting more activate cell proliferation (*P *<* *0.05). There were no notable differences in OD value among the blank, NC, and miR‐92a inhibitor + siRNA‐PTEN groups at any time points (*P *>* *0.05). The OD value of the miR‐92a inhibitor and normal groups was lower than that of the blank group at all the time points, especially notable at 96 h (*P *<* *0.05). And, no obvious difference was observed between the miR‐92a inhibitor and normal groups at any time points (*P *>* *0.05) (Fig. 5 and Table A2). These findings suggest that the overexpression of miR‐92a may promote the proliferation of cervical cancer cells.

**Figure 5:** Cell proliferation at the point of 24 h, 48 h, 72 h, and 96 h in seven groups after transfection. *, *P *<* *0.05 compared with the blank and negative control groups.

### MiR‐92a inhibits cell apoptosis in vitro

Flow cytometry was adopted in order to identify cell apoptosis, and results revealed that cell apoptosis rate was higher in the normal group compared to the other six groups (*P *<* *0.05). No obvious differences in terms of cell apoptosis rate were found among the blank, NC, miR‐92a inhibitor + siRNA‐PTEN groups (*P *>* *0.05). Compared with the blank and NC groups, an increased cell apoptosis rate was found in the miR‐92a inhibitor group, while a decreased apoptosis rate was observed in the miR‐92a mimic and siRNA‐PTEN groups. No such significant differences were found between the miR‐92a mimic and siRNA‐PTEN groups (*P *>* *0.05) (Fig. 6 and Table A3). Taken together, these results suggest that overexpressed miR‐92a inhibits apoptosis in cervical cancer cell.

**Figure 6:** Cell apoptosis in seven groups after transfection. (A) cell apoptosis in seven groups; (B) apoptosis rate in seven groups; *, *P *<* *0.05 compared with the normal group; ^#^, *P *<* *0.05 compared with the blank and negative control groups.

### MiR‐92a arrests the cell number in the S phase in vitro

According to the flow cytometry results, the cell cycle presented no remarkable differences among the blank, NC, and miR‐92a inhibitor + siRNA‐PTEN groups (*P *>* *0.05). Compared with the normal group, a higher number of cells were found to be arrested in the S phase while less in the G0/G1 phase in all other six groups (*P *<* *0.05). The cell number was arrested in the S phase, and was lower in the G0/G1 phase in the miR‐92a mimic and siRNA‐PTEN groups in comparison with the blank and NC groups, while the miR‐92a inhibitor group followed opposite trends (all *P *<* *0.05). There were no significant differences in terms of cell cycle between the miR‐92a mimic and siRNA‐PTEN groups (*P *>* *0.05). It indicated that overexpressed miR‐92a could promote cell proliferation. No obvious differences were found in the number of cells in the G2/M phase in all seven groups (*P *>* *0.05) (Fig. 7 and Table A4). These results suggest that miR‐92a enhances cell proliferation.

**Figure 7:** Changes in cell cycle distribution in seven groups after transfection. (A) cell cycle under microscope; (B) comparison of cell cycle among seven groups; *, *P *<* *0.05 compared with the normal group; ^#^, *P *<* *0.05 compared with the blank and negative control groups.

### Overexpressed miR‐92a increases levels of TNF‐*α* and sIL‐2R in vitro

The results of ELISA indicated that compared with the normal group, TNF‐*α* and sIL‐2R levels were significantly increased in the other six groups (*P *<* *0.05). As opposed to the blank and NC groups, the levels of TNF‐*α* and sIL‐2R were remarkably elevated in the miR‐92a mimic and siRNA‐PTEN groups, while declined in the miR‐92a inhibitor group (*P *<* *0.05). The levels of TNF‐*α* and sIL‐2R in the miR‐92a mimic group were higher compared to the miR‐92a inhibitor group (*P *<* *0.05). No significant differences were observed between the miR‐92a mimic and siRNA‐PTEN groups and among the blank, NC and miR‐92a inhibitor + siRNA‐PTEN groups (*P *>* *0.05) (Fig. 8). In conclusion, overexpressed miR‐92a increases the levels of TNF‐*α* and sIL‐2R.

**Figure 8:** TNF‐*α* and sIL‐2R levels in seven groups after cell transfection detected by ELISA. TNF‐*α*, tumor necrosis factor‐*α*; sIL‐2R, soluble interleukin‐2 receptor; *, *P *<* *0.05 compared with the normal group; ^#^, *P *<* *0.05 compared with the blank and negative control groups.

### Transplanted tumor volume increases in the mice transfected with miR‐92a mimic

Based on the transplanted tumor assay, after the first three injections (at 0th day, 3th day, and 6th day, respectively), there was no significant difference in terms of tumor growth among the seven groups. After the last three injections (at 9th day, 12th day, and 15th day), the size of the tumor grew bigger in the miR‐92a mimic group compared to the blank and NC groups, and part of tumor metastasis was found in the forelimb and abdomen. In contrast, tumor growth was restricted in the miR‐92a inhibitor group with smaller in situ tumors and unnoticeable metastatic tumor nodules. Compared with the other groups, the tumor volume in the miR‐92a inhibitor group was the smallest (Fig. 9). These findings provide evidence that transplanted tumor elevated markedly in the mice transfected with miR‐92a mimic.

**Figure 9:** Tumor volume of nude mice after transfection in seven groups. *, *P *<* *0.05 compared with the blank and negative control groups.

## Discussion

Cervical cancer currently presents as the leading cause of female’ deaths in childbearing age, and existing conventional therapy screening methods remain ineffective for advanced stage cervical cancer and inaccessible to developing regions 18; thus, cervical cancer and factors affecting it need to be unearthed in order to explore new approaches and improve the quality of life. This study aims to explore the effects of miR‐92a on tumor growth and immune function of cervical cancer by targeting PTEN *via* the MAPK/ERK signaling pathway in U14 cervical cancer mouse models.

Firstly, we observed a decreased mRNA and protein expression of PTEN and increased miR‐92a expression, mRNA and protein expressions of ERK1 and ERK2 in the U14 cervical cancer tissue. The tumor‐suppressed protein PTEN is common in human cancer and infrequently found in cervical cancer and even lower in advanced stage compared to the early stages 19. ERK1 and ERK2 are associated with protein‐serine kinases, and are a part of the Ras‐Raf‐MEK‐ERK signal transduction cascade, which participates in various cell processes 20. A previous study demonstrated that ERK1 and ERK2 were highly expressed in cervical cancer, which was in line with our results 13. In addition, miR‐92a was also indicated to be up‐regulated in invasive cervical cancer tissue, with higher expression related to a higher grade of cancer 9. These data elucidate the role played by miR‐92a, PTEN, ERK1, and ERK2 in the progression of cervical cancer and gives us insight into the interaction among the above molecules during cervical cancer progression. In addition, our results showed that U14 cervical cancer tissue had higher serum TNF‐*α* and sIL‐2R levels. TNF‐*α*, a Th1 proinflammatory cytokine, has been proven to play a significant role in the process of tumor necrosis and in cervical cancer progression 21. A previous study also demonstrated that serum proteins such as sTNFRI and sTNFRII were found to be markedly increased in cervical cancer with tumor‐promoting stage 22. Thus, elevated levels of serum TNF‐*α* and sIL‐2R suggest the more severe condition of cervical cancer.

Our results show that the cells transfected with miR‐92a mimic exhibited a lower expression of PTEN but higher expression of ERK1 and ERK2 compared with the blank group. In a previous study, a decreased expression of PTEN and an increased expression of miR‐92a were found in colorectal cancer tissues, suggesting a negative correlation 23. It was also demonstrated that miR‐92a participates in the regulation of cell growth, migration, and invasion in the SW480 cells although the inhibition of PTEN expression 24. Moreover, miR‐17‐92 cluster, involving miR‐92a and some other miRNAs, has been previously indicated in inducing continuous activation of ERK1/2 signaling in DU145 prostate cancer cells 25. In the progression of other cancers such as prostate cancer, PTEN loss can stimulate the activity of the MAPK pathway, in both primary and advanced stages of lesions 26. It has been reported that PTEN was involved in the regulation of several signaling pathways, including the ERK1/2 pathway, and its activation typically results in cancer development and progression 27. Besides, high levels of serum TNF‐*α* and sIL‐2R levels were detected in cells transfected with miR‐92a mimic. In the progression against pathogens, miR‐92a mimics were evidenced to induce the production of TNF‐*α* according to a previous research 28. Furthermore, a previous study proved that overexpressed miR‐155, another miRNA, inhibited levels of interleukin‐2 (IL‐2) 29.

In addition, we revealed that the proliferation of cervical cancer cell was accelerated in cells transfected with miR‐92a mimic or siRNA against PTEN, but apoptosis was inhibited *via* the activation of the MAPK/ERK signaling pathway. It has been confirmed that miR‐92a plays a key role as an oncogene in order to promote cell proliferation by targeting FBXW7 in gastric cancer 30. Similarly, the up‐regulated miR‐92a in lung cancer cells was a promoting factor for cell proliferation but acts as an inhibitor for cell apoptosis 30. In contrast, the inhibition of miR‐92a can significantly decrease cell growth and induce apoptosis, which was assessed in a previous study 31. Correspondingly, a previous study found that up‐regulated PTEN suppressed colorectal cancer cell proliferation and induced apoptosis, which suggested that down‐regulation of PTEN may deliver opposite results 32. These aforementioned evidences and findings reveal the role of miR‐92a overexpression and PTEN silencing in cervical cancer cell function.

In summary, our study provides evidences stating that up‐regulation of miR‐92a can promote cervical cancer cell proliferation and suppress the immune function by targeting PTEN by activating the MAPK/ERK signaling pathway. Our conclusion can be further researched and studied in order to achieve the clinical potential of miR‐92a in the treatment of cervical cancer and raising the quality of life.

## Conflict of Interest

None.

## Appendix

**Table A1:** The miR‐92a expression and mRNA and protein expressions of PTEN, TNF‐*α*, sIL‐2R, ERK1, and ERK2 after cell transfection in seven groups

	Normal	Blank	NC	miR‐92a mimic	miR‐92a inhibitor	siRNA‐PTEN	miR‐92a inhibitor + siRNA‐PTEN	*P*
mRNA								
miR‐92a	0.997 ± 0.045	2.347 ± 0.089*	2.403 ± 0.084*	4.539 ± 0.468*#	1.574 ± 0.039*#	2.098 ± 0.084*	2.278 ± 0.040*	<0.001
PTEN	1.018 ± 0.053	0.439 ± 0.036*	0.450 ± 0.037*	0.193 ± 0.021*#	0.762 ± 0.079*#	0.252 ± 0.013*#	0.481 ± 0.044*	<0.001
ERK1	0.989 ± 0.048	2.107 ± 0.092*	2.196 ± 0.109*	3.175 ± 0.302*#	1.485 ± 0.098*#	3.007 ± 0.268*#	1.989 ± 0.156*	<0.001
ERK2	1.005 ± 0.060	1.858 ± 0.098*	2.008 ± 0.090*	2.803 ± 0.281*#	1.442 ± 0.085*#	2.791 ± 0.179*#	1.896 ± 0.121*	<0.001
TNF‐a	1.017 ± 0.059	1.789 ± 0.104*	1.757 ± 0.089*	2.709 ± 0.176*#	1.392 ± 0.097*#	2.693 ± 0.180*#	1.795 ± 0.112*	<0.001
SIL‐2R	0.973 ± 0.033	2.267 ± 0.158*	2.336 ± 0.180*	3.378 ± 0.218*#	1.583 ± 0.139*#	3.206 ± 0.298*#	2.209 ± 0.207*	<0.001
Protein								
PTEN	1.273 ± 0.042	0.742 ± 0.044*	0.706 ± 0.065*	0.221 ± 0.074*#	0.937 ± 0.057*#	0.246 ± 0.072*#	0.653 ± 0.097*	<0.001
ERK1	0.217 ± 0.030	0.783 ± 0.043*	0.801 ± 0.045*	1.573 ± 0.063*#	0.421 ± 0.069*#	1.474 ± 0.058*#	0.827 ± 0.056*	<0.001
ERK2	0.209 ± 0.025	0.763 ± 0.042*	0.806 ± 0.051*	1.480 ± 0.086*#	0.397 ± 0.023*#	1.376 ± 0.081*#	0.819 ± 0.078*	<0.001
p‐ERK1/2	0.231 ± 0.024	0.894 ± 0.095*	0.922 ± 0.103	1.191 ± 0.089*#	0.453 ± 0.052*#	1.145 ± 0.086*#	0.795 ± 0.078*	<0.001

**P *<* *0.05 compared with the normal group; ^#^ *P *<* *0.05 compared with the blank and negative control groups.

**Table A2:** The effect of transfected groups on the growth of U14 cervical cancer cells detected by CCK‐8 assay

	Normal	Blank	NC	miR‐92a mimic	miR‐92a inhibitor	siRNA‐PTEN	miR‐92a inhibitor + siRNA‐PTEN
24 h	0.21 ± 0.01	0.24 ± 0.01	0.24 ± 0.01	0.24 ± 0.02	0.21 ± 0.01	0.24 ± 0.01	0.24 ± 0.02
48 h	0.30 ± 0.03	0.38 ± 0.03	0.37 ± 0.02	0.37 ± 0.04	0.32 ± 0.02	0.37 ± 0.03	0.38 ± 0.04
72 h	0.36 ± 0.03*	0.48 ± 0.02	0.47 ± 0.04	0.61 ± 0.03*	0.38 ± 0.03*	0.59 ± 0.02*	0.50 ± 0.03
96 h	0.40 ± 0.06*	0.58 ± 0.03	0.55 ± 0.05	0.73 ± 0.05*	0.42 ± 0.05*	0.69 ± 0.06*	0.60 ± 0.05

*P *<* *0.05 compared with the blank and negative control groups.

**Table A3:** The effect of transfected groups on the apoptosis of U14 cervical cancer cells

Normal	Blank	NC	miR‐92a mimic	miR‐92a inhibitor	siRNA‐PTEN	miR‐92a inhibitor + siRNA‐PTEN	P
12.56 ± 0.63	4.97 ± 0.49*	5.10 ± 0.45*	2.43 ± 0.43*#	8.79 ± 0.30*#	2.57 ± 0.19*#	5.19 ± 0.21*	<0.001

**P *<* *0.05 compared with the normal group; ^#^ *P *<* *0.05 compared with the blank and negative control groups.

**Table A4:** The effect of transfected groups on the cell cycle of U14 cervical cancer cells

	Normal	Blank	NC	miR‐92a mimic	miR‐92a inhibitor	siRNA‐PTEN	miR‐92a inhibitor + siRNA‐PTEN
G0/G1	72.56 ± 1.63	59.97 ± 2.09*	60.30 ± 0.75*	48.43 ± 1.23*#	68.79 ± 1.30*#	49.07 ± 1.19*#	60.85 ± 0.50*
S	16.30 ± 0.51	27.58 ± 1.09*	27.00 ± 1.03*	39.69 ± 1.21*#	21.09 ± 0.28*#	38.21 ± 0.86*#	26.96 ± 0.69*
G2/M	11.14 ± 1.62	12.45 ± 1.11	12.70 ± 1.41	11.88 ± 1.16	10.12 ± 1.56	12.72 ± 1.63	12.19 ± 0.94

**P *<* *0.05 compared with the normal group; ^#^ *P *<* *0.05 compared with the blank and negative control groups.
